The article "COVID-19 Semantic Pneumonia Segmentation and Classification Using Artificial Intelligence" was retracted in 2025. Reasons: signs of a paper mill; suspected computer-generated content; unreliable results or conclusions; concerns about the data.

# COVID-19 Semantic Pneumonia Segmentation and Classification Using Artificial Intelligence

**DOI:** 10.1155/2022/5297709

**Published:** 2022-09-15

**Authors:** Mohammed J. Abdulaal, Ibrahim M. Mehedi, Abdullah M. Abusorrah, Abdulah Jeza Aljohani, Ahmad H. Milyani, Md. Masud Rana, Mohamed Mahmoud

**Affiliations:** ^1^Department of Electrical and Computer Engineering (ECE), King Abdulaziz University, Jeddah, Saudi Arabia; ^2^Center of Excellence in Intelligent Engineering Systems (CEIES), King Abdulaziz University, Jeddah, Saudi Arabia; ^3^Department of Electrical and Electronic Engineering, Rajshahi University of Engineering and Technology (RUET), Rajshahi, Bangladesh; ^4^Electrical and Computer Engineering Department, Tennessee Technological University, Cookeville, TN, USA

## Abstract

Coronavirus 2019 (COVID-19) has become a pandemic. The seriousness of COVID-19 can be realized from the number of victims worldwide and large number of deaths. This paper presents an efficient deep semantic segmentation network (DeepLabv3Plus). Initially, the dynamic adaptive histogram equalization is utilized to enhance the images. Data augmentation techniques are then used to augment the enhanced images. The second stage builds a custom convolutional neural network model using several pretrained ImageNet models and compares them to repeatedly trim the best-performing models to reduce complexity and improve memory efficiency. Several experiments were done using different techniques and parameters. Furthermore, the proposed model achieved an average accuracy of 99.6% and an area under the curve of 0.996 in the COVID-19 detection. This paper will discuss how to train a customized smart convolutional neural network using various parameters on a set of chest X-rays with an accuracy of 99.6%.

## 1. Introduction

The emerging COVID-19 pandemic continues to threaten global health, the economy, and quality of life. According to the World Health Organization (WHO), it is worth noting that this disease was first detected in late 2019 in Wuhan, China, and then spread to the rest of the world, leading to its classification as a pandemic. The current confirmed cases of this disease exceed 140 million cases, and the number of deaths is 3 million confirmed cases [1]. There are nearly 600,000 confirmed cases in the world within one week, and this number is large compared to the rest of the endemic diseases in the world. It is worth noting that the number of injured and recovered patients without being recorded is double this number [1–5].

This led to the imposition of restrictions and a complete closure on travel, global trade, and movement to reduce the number of injuries, which led to the deterioration of the gigantic and emerging economies. The COVID-19 virus consists of more than one strain and develops gradually, making it difficult to discover and develop an effective vaccine for eradicating this disease so far [2]. All this led to researchers' participation in various parts of the world to establish rapid systems for early detection and isolation of infections to reduce the disease's spread and control it and return life to what it was before the pandemic. Therefore, early and accurate detection of pneumonia, blood clots, and severe acute respiratory syndrome associated with SARS-CoV-2 is the focus of the world's attention and is one of the most pressing issues at the moment. There are three different methods of detecting the disease inside hospitals and laboratories, such as blood analysis, x-rays, medical imaging, and other traditional methods that lead to an increase in the number of injuries between doctors and nurses through patients' movement through different hospitals [3]. Therefore, early, accurate, and electronic remote detection is essential. The primary indicators of early diagnosis of this disease are lung injury and blood clotting, as it causes difficulty breathing and blood clotting. Therefore, there are many challenges associated with this field, which can be summarized as follows [6–12]:

1. Chest X-ray (CXR) image contains a wide variability and a diversity of features [3].
2. The diagnosis of any disease depends on linking symptoms together and extracting semantic features in real time. Therefore, any diagnostic system requires high speed and accuracy in performing the tasks [13].
3. The classification and prediction processes using machine leaning algorithms may suffer from overfitting problems [14].

The article "COVID-19 Semantic Pneumonia Segmentation and Classification Using Artificial Intelligence" was retracted in 2025. Reasons: signs of a paper mill; suspected computer-generated content; unreliable results or conclusions; concerns about the data.

Also, some common symptoms such as high fever, severe fatigue, and dry cough were reported in some confirmed cases of COVID-19 [1]. Hence, these symptoms can help us diagnose COVID-19 at an early stage. We will first use the blood vessel clot to distinguish between bacterial pneumonia, COVID-19, and a healthy lung. The main contributions of this paper are as follows:

  (1) Conducting a thorough analysis of the studies related to early detection of COVID-19 and comparing them with our proposed model.
  (2) A proposed model was made to differentiate between cases infected with SARS-COV-2 or COVID-19 and bacterial pneumonia and the normal cases. The model was developed using artificial intelligence techniques and a pretrained deep learning network for accurate and rapid injury cases.
  (3) Feature extraction techniques were used to segment the affected regions.
  (4) More than one set of data was used from different sources and divided into learning and testing data using 10-fold cross-validation to refine the deep learning network and overcome overfitting problems.

The article "COVID-19 Semantic Pneumonia Segmentation and Classification Using Artificial Intelligence" was retracted in 2025. Reasons: signs of a paper mill; suspected computer-generated content; unreliable results or conclusions; concerns about the data.

The remainder of this article will be divided into the following parts. Related works will be discussed in Section 2. The proposed framework and algorithms will be discussed in Section 3. The results of different experiments will also be discussed and compared with other similar studies in Section 4. Finally, the various conclusions will be presented in Section 5.

## 2. Related Works

We will review the different efforts of researchers from various prestigious scientific journals and the different methods and patterns of artificial intelligence that they have found for early detection of the emerging coronavirus disease as summarized in Table 1. Unfortunately, there are different traditional methods for predicting, detecting, and responding to this disease based on knowledge of the places most affected by heart disease and diabetes. In addition to the understanding of population density and social distancing, methods were used to detect and predict the COVID-19. However, all these traditional methods do not lead to a decrease in the rate of injuries and deaths [21–23]. Therefore, artificial intelligence methods and deep learning outcomes have an important role in early detection and isolation of affected cases in a fast and inexpensive way [5, 24].

It has been noted in most international research that the disease can be detected through a chest X-ray or a CT scan [4, 25, 26]. However, detection by means of a CT scan is more expensive than a CXR, but it is characterized by its accuracy. Therefore, the main challenge here is to raise the level of accurate detection through x-rays to be like a CT scan. It has also been observed that the disease can be detected by detecting peripherally distributed pneumonia that represents vitreous opacity and vascular thickening. However, this method may have a low accuracy rate if the extracted feature is not on the affected place, and this is what will be emphasized in our paper. Convolutional neural networks (CNNs) are widely used in medical imaging and disease detection. In this paper, we review the latest research contributions of deep learning application to detect COVID-19 from CXR images, highlight the challenges involved, and identify future investigations required [27, 28].

Zhao et al. [29] proposed the traditional deep learning neural network on a dataset of 275 chest X-rays to classify the images as normal or contain pneumonia. However, the accuracy of this method was very weak, as it was only 85% accurate. Maghdid et al. [30] proposed a preassigned AlexNet model to classify the CXR images as normal or contain pneumonia due to SARS-COV-2 with an accuracy of 94.1%. But the problem with this research is that it depends on a prior model and can be affected by overfitting and cannot extract the affected patterns only. Also, this model's accuracy is still poor, although it is higher than the previous research.

The article "COVID-19 Semantic Pneumonia Segmentation and Classification Using Artificial Intelligence" was retracted in 2025. Reasons: signs of a paper mill; suspected computer-generated content; unreliable results or conclusions; concerns about the data.

Bukhari et al. [27] relied on a previously assigned ResNet-50 form to detect CXR images as natural or contain pneumonia due to SARS-COV-2 with an accuracy of 98%. But the problem with this research is that it depends on a prior model as well. The deep web has been trained on a small number of images, and it can be affected by the overfitting problem. Although the model's accuracy is considered relatively high, it cannot be relied upon entirely in early diagnosis. Santosh et al. [15] introduced a network powered by Truncated Inception technology to classify CXR-positive images from normal states. They also used different data sets with an accuracy of 99%. But the main problem with this work is that it has nonclinical effects that are performed.

Pereira et al. [31] presented a proposal for hierarchical classification of CXR images and to detect whether they are normal or contain pneumonia depending on the hierarchy of different patterns and the training of a pretrained CNN network for this purpose. They also used reconfiguration algorithms to solve the problem of data imbalance. With these two methods, they were able to achieve an accuracy level of 89%. Despite its efficiency, this system's accuracy needs to be improved and it needs to be applied to a larger number of images. Ozturk et al. [16] proposed a novel method for accelerating the identification of COVID-19 disease using CXR images. Their schema obtained a classification efficiency of 98% and 87.02% for dual and multilayer classification, respectively. This research's problem lies in the technique's weakness for multilayer classification and the time consumed for the classification is relatively high. Ucar and Korkmaz [9] proposed an innovative paradigm for quick analysis of SARS-COV-2 based on Deep Bayes-Squeeze Network technology. Their model achieved an accuracy rate of 98.3% for multiple classes. Despite its relatively high accuracy, the main problem with this research is that the time consumed for classification is relatively high.

Abdel Moneim et al. [32] previously customized a deep learning neural network model based on Resnet-50 to classify CXR images using 10-fold validation and the result was 97.28% accuracy. But the problem with this research is that it depends on a prior model that takes a long time to train because of the lack of focus on the affected area only. Also, the accuracy of this model is still unreliable because it is trained on a small data set, although it is relatively high. Şengür et al. [19] suggested a CNN schema based on preassigned Resnet-50 and SVM with linear core function to classify CXR images and obtained an efficiency of 94.7%. However, the problem with this research is that they used an insufficient amount of CXR images. Therefore, a recommendation to run the model on a more significant number of unbalanced data is required. The accuracy rate is still not satisfactory. Hassibi et al. [13] improved the generalization model for CNN and speeded up the network by selecting the extracted patterns using the second derivative in the Taylor series. This resulted in a 34% decrease in network parameters and improved mass classification performance. Rajaraman et al. [33] proposed a new custom CNN of ImageNet pretrained models on CXR collections. To improve performance, their method combines knowledge transfer with iterative model pruning and ensemble learning. Consequently, they achieved an accuracy rate of 99%. Chen et al. [34] presented two collaborative networks capable of analyzing CXR images with multiple segmentation labels based on lung segmentation. AUC of 0.82 was achieved using the proposed self-adaptive weighted approach. Elzeki et al. [20] developed a Chest X-ray COVID Network (CXRVN) using three distinct CXR datasets. CXRVN along with GAN achieved 96.7% accuracy.

The article "COVID-19 Semantic Pneumonia Segmentation and Classification Using Artificial Intelligence" was retracted in 2025. Reasons: signs of a paper mill; suspected computer-generated content; unreliable results or conclusions; concerns about the data.

## 3. Proposed Framework and Methods

In this section, the different stages of the proposed model will be explained.  Figure 1 shows the proposed framework. The proposed model contains two serial stages. The first stage includes various preprocessing tasks such as filtering, adaptive histogram equalization, and semantic segmentation. Thereafter, classification and detection of infected subjects are achieved using pretrained CNN model. Finally, it classifies the given subject as normal, bacterial pneumonia, or COVID-19.

### 3.1. Preprocessing Phase

This phase takes the standard dataset as input and produces the segmented lungs as output.  Figure 2 shows the main subphases of this stage. Algorithm 1 shows the preprocessing steps [35, 36].

(1) Input dataset includes two datasets of CXR images with 1024 × 1024 and 512 × 512 pixel resolution from different sources [37, 38]. The dataset was released for the different sources. The acquisition dataset involves natural and abnormal CXR images with normal and COVID-19 pneumonia.
(2) Gray scale conversion: this subphase converts the RGB image into gray scale level. Based on the probability theory, the dynamic adaptive histogram equalization obtains the gray mapping of pixels to uniform and smooth gray levels [39].  Figure 3 represents sample of original images including the normal and abnormal CXR.
(3) Adaptive histogram equalization (AHE): if *n* is the number of gray levels obtained in the original image, *p* is the number of pixels in the image with kth gray level, and *T* is the whole number of pixels in the image. AHE is computed according to Equation (1).  Figure 4 represents a sample of enhanced images after applying the AHE to every image in the dataset. Consider the following:
  (1) $$\begin{array}{c} {\text{AHE}}_{i}=\left(m-1\right)\sum_{k=0}^{i}\frac{p_{i}}{T}. \end{array}$$
(4) Semantic Segmentation: Deeplabv3plus is a model that segments images and obtains semantic labels based on deep learning architecture.  Figure 5 represents DeepLabv3Plus architecture.

The article "COVID-19 Semantic Pneumonia Segmentation and Classification Using Artificial Intelligence" was retracted in 2025. Reasons: signs of a paper mill; suspected computer-generated content; unreliable results or conclusions; concerns about the data.

### 3.2. Deep CNN for COVID-19 Classification (DCNCC) Phase

This phase is the essential part of our proposed model to build a new innovative structure to classify the chest X-ray images of COVID-19 to determine the typical images and the abnormal images. The standard dataset is divided into training and testing datasets with 70% and 30%, respectively. The data augmentation process is performed on the training dataset before applying the DCNCC phase with 10-fold cross-validation to avoid overfitting problems. This complex neural network is the first innovative network specialized in image segmentation and analysis of COVID-19 CXR. The proposed model (DCNCC) architecture is represented in Figure 6. The proposed deep neural network consists of three wrapping layers, three collocation layers, and one fully interconnected layer. Data augmentation represented in Figure 5 is a regularization procedure that produces a tremendous volume of practical units through applying various conversions such as rotating, resizing, flipping, shifting, and changing the brightness conditions. Transfer learning concept is based on description learning with the underlying premise that some patterns are common to several various tasks. In Figure 5, we use 256*∗*256 processed training CXR size to enter the semantic convolutional network. Also, we use three convolutional blocks. Each block includes a batch normalization, ReLU activation function, Max pooling, Dropout and Flatten. The rectified linear unit (ReLU) is used as the hidden layers to allow faster learning.

ReLU has a great advantage over sigmoid and tanh. We use hybrid optimization algorithms: Butterfly Optimization Algorithm (BOA), particle swarm optimization (PSO), and modified salp swarm algorithm (SSA).  Figure 7 represents the steps of creating DCNCC (Algorithm 2) layers and network.  Table 2 shows the overall parameters used in the proposed DCNCC training network. The iterative pruning model was used to reduce complexity and time consumed to obtain the optimum number of neurons, and the performance efficiency was not compromised. We used the average ratio of zeros (APoZ) with an abnormal CXR. Algorithm 3 shows the iterative pruning of Net steps.

The article "COVID-19 Semantic Pneumonia Segmentation and Classification Using Artificial Intelligence" was retracted in 2025. Reasons: signs of a paper mill; suspected computer-generated content; unreliable results or conclusions; concerns about the data.

## 4. Experimental Results Setup

In this section, the practical experiments will be explained. Firstly, the type and size of the data used will be described. Secondly, the results of each trial experiment will be presented and discussed. Finally, comparisons between the proposed model and the rest of the relevant models will be explained. The experiments of this research were carried out using two tools. Firstly, MATLAB version 2021, Intel Core i7 CPU, and 8 GB RAM were used to perform semantic segmentation. Secondly, Google Cola, Tensor Processing Unit (TPU), and 32 GB RAM were used to perform data augmentation, pruning, and deep learning processes.

### 4.1. Dataset Characteristics

Experiments were carried out on two types of datasets, as shown in Table 3. The first dataset (DS1) contains two classes (positive and negative labels). DS1 has 15264 images of the training process and 400 images of the testing process. The second dataset (DS2) contains three classes (COVID-19 pneumonia, bacterial pneumonia, and normal labels). DS2 has 1811 images of the training process and 484 images of the testing process.  Table 4 represents the configuration parameters used in training process [40].

### 4.2. Model Evaluation

#### 4.2.1. Evaluation Metrics

We use four metrics to evaluate the proposed framework. These metrics are sensitivity, specificity, accuracy, and f-measure. These measurement equations are used as follows:

(2) $$\begin{array}{c} \text{SN}=\frac{\text{TP}}{\text{TP}+\text{FN}},\\ \text{SP}=\frac{\text{TN}}{\text{TN}+\text{FP}},\\ \text{AC}=\frac{\text{TP}+\text{TN}}{\text{TP}+\text{TN}+\text{FP}+\text{FN}},\\ F1-S=\frac{\text{TP}}{\text{TP}+1/2\left(FP+FN\right)}, \end{array}$$

where TP = True Positive, FN = False Negative, FP = False Positive, and TN = True Negative.

#### 4.2.2. Experimental Results

*(1) First Experiment*. In the first experiment, pretrained networks such as ResNet 50 with many epochs (20, 30, 40, 50, and 60) and without data augmentation are conducted with 500 extracted features. In this experiment, we found that 50 epochs resulted in the highest accuracy (92.3%) and that 60 epochs resulted in a decrease in accuracy due to overtraining.

*(2) Second Experiment*. In the second experiment, data augmentation to increase size of data and pretrained networks (ResNet 50 and DenseNet) with 1000 extracted features are conducted but without semantic segmentation. In this experiment, we found that 50 epochs resulted in the highest accuracy (95.1%).

*(3) Third Experiment*. In the third experiment, data augmentation, pretrained networks (ResNet 50 and DenseNet) with 1200 extracted features, and semantic segmentation using Deeplabv3Plus are applied but without pruning. In this experiment, we found that 50 epochs resulted in the highest accuracy (96.6%).

*(4) Last Experiment*. In the last experiment, data augmentation, pretrained networks (ResNet 50 and DenseNet) with 1000 extracted features, semantic segmentation using Deeplabv3Plus, and data pruning are applied. In this experiment, we found that 50 epochs resulted in the highest accuracy (99.6%).

The article "COVID-19 Semantic Pneumonia Segmentation and Classification Using Artificial Intelligence" was retracted in 2025. Reasons: signs of a paper mill; suspected computer-generated content; unreliable results or conclusions; concerns about the data.

## 5. Discussion

We conducted four experiments to find more rapid, robust, and accurate training and classification configuration factors. Datasets are divided into 70% for training and 30% for testing. We use 10-fold cross-validation to avoid overfitting problems. Data augmentation is used to increase size of data and overcome unbalanced data. In the first experiment, pretrained networks such as ResNet 50 with many epochs (20, 30, 40, 50, and 60) and without data augmentation are conducted with 500 extracted features. In this experiment, we found that 50 epochs resulted in the highest accuracy (92.3%) and that 60 epochs resulted in a decrease in accuracy due to overtraining. In the second experiment, data augmentation to increase size of data and pretrained networks (ResNet 50 and DenseNet) with 1000 extracted features are conducted but without semantic segmentation. In this experiment, we found that 50 epochs resulted in the highest accuracy (95.1%). In the third experiment, data augmentation, pretrained networks (ResNet 50 and DenseNet) with 1200 extracted features, and semantic segmentation using Deeplabv3Plus are applied but without pruning. With 50 epochs, we were able to achieve the highest accuracy of 96.6%. In order to achieve the highest accuracy, pretrained networks (i.e., ResNet 50 and DenseNet) with 1000 extracted features were used that have achieved 99.6% accuracy. We analyzed and enumerated the model's performance during the learning phase. We used traditional measurement methods such as Sensitivity (SN), Specificity (SP), Accuracy (AC), and F1-score (*F*1–S) to measure the model's efficiency.  Figure 8 represents the detailed confusion matrix for DS1 and DS2. Tables 5 and 6 summarized the Sensitivity (SN), Specificity (SP), Accuracy (AC), and *F*1-score (*F*1–S) for DS1 and DS2 using (RESNET-50+ DenseNet), respectively.  Figure 9, Figure 10, and Figure 11 showed the training and validation accuracy and loss, respectively, using 50 epochs with 700 iterations.

The article "COVID-19 Semantic Pneumonia Segmentation and Classification Using Artificial Intelligence" was retracted in 2025. Reasons: signs of a paper mill; suspected computer-generated content; unreliable results or conclusions; concerns about the data.

In each experiment, a new technique, such as data augmentation, hybrid CNN, semantic segmentation, and data pruning, was added to increase the number of distinct features, which can increase the accuracy of the diagnosis. But it increases the time consumption. So, we use semantic segmentation to find Region of Interest (ROI) to decrease time consumption. In Table 7, we found that the proposed method achieved the highest accuracy rate, but it still consumes some additional time. A comparison was made between the average of our experiments and the results of others. In Table 7 and Figure 12, the statistical average is shown between the proposed model and the rest of the modern models that discuss the same issue. We clearly found that the proposed model provided the highest accuracy and shortest time consumption as shown in Table 7 and Figure 12.

Overall, the proposed model outperformed the competitive models, but the hyperparameters of the proposed models were selected on trial-and-error basis. Therefore, in the near future, we will use different parameters optimization techniques [21–23, 41–43] to automatically select the hyperparameters. Additionally, ensembling of the models [44–46] can be achieved to overcome the overfitting problem. [47].

## 6. Conclusions

In this article, we build a proposed model called DCNCC to classify and detect CXR images of COVID-19. The proposed model was worked out in two stages. The first stage is optimizing the images by using dynamic adaptive histogram equalization, semantic segmentation using DeepLabv3Plus, and augmenting data by flipping horizontally, rotating, and flipping vertically. The second stage builds a custom CNN model by using several pretrained ImageNet models and comparing them to repeatedly trim the best-performing models to reduce complexity and improve memory efficiency. For COVID-19 detection, the proposed model achieved an average accuracy of 99.6% and an area under the curve of 0.996, respectively.

## Figures and Tables

**Figure 1:** The Proposed Framework.

**Figure 2:** Main subphases in preprocessing stages.

**Figure 3:** Original images: (a) normal CXR, (b) COVID-19 pneumonia CXR.

**Figure 4:** Enhanced images using adaptive histogram equalization: (a) normal CXR, (b) COVID-19 pneumonia CXR.

**Figure 5:** Deeplabv3Plus architecture.

**Figure 6:** Proposed DCNCC model.

**Figure 7:** DCNCC architecture.

**Figure 8:** (a) Confusion matrix of the first experiment using DS1. (b) Confusion matrix of the second experiment using DS2.

**Figure 9:** Training and validation accuracy curve for proposed model using RESNET-50+ DenseNet, 700 iterations and 50 epochs.

The article "COVID-19 Semantic Pneumonia Segmentation and Classification Using Artificial Intelligence" was retracted in 2025. Reasons: signs of a paper mill; suspected computer-generated content; unreliable results or conclusions; concerns about the data.

**Figure 10:** Training and validation loss curve for proposed model using RESNET-50+ DenseNet, 700 iterations and 50 epochs.

**Figure 11:** Validation accuracy curve against validation loss curve for proposed model using RESNET-50+ DenseNet, 700 iterations and 50 epochs.

**Figure 12:** Accuracy chart between proposed model and related works.

**Algorithm 1:** Preprocessing Configurations.

**Algorithm 2:** DCNCC Architecture.

**Algorithm 3:** Pruned Net

**Table 1:** Summary of the related works.

Ref.	A	Results (%)	Limitations
[15]	Truncated inception network	98.5	(i) Limited dataset is used.
			(ii) In stacking, the original dimensions are solved.
			(iii) Images and the structured images must be the same.

[16]	DarkCovidNet	87.02	(i) End-to-end architecture.
			(ii) Manual feature extraction.
			(iii) Including a severely low number of image samples.
			(iv) Imprecise localization on the chest region

[9]	Bayes-SqueezeNet	97.9	(i) This study is conducted on a publicly dataset, which contains less than 100 COVID-19 images, and more than 5,000 non-COVID images. Due to the limited number of COVID-19 images publicly available so far, further experiments are needed on a larger set of cleanly labeled COVID-19 images for a more reliable estimation of the sensitivity rates.
[17]	DenseNet	85	(ii) Limited dataset is used.
[18]	MobileNet	94.7	—

[19]	Resnet-50+SVM	94.7	(i) The limitation of this methodology is that if the patient is in a critical situation and unable to attend for Xray scanning.
			(ii) Small dataset.
			(iii) Authors involved SARS&MER cases in COVID positive classes.

[20]	CXRVN	97.5	(i) Time consuming.
			(ii) Lack of extract semantic reliable features.
			(iii) Binary classifier.

**Table 2:** Proposed model parameters for training process.

Parameters	Values	Parameters	Values
Input size	256^*∗*^256	Pool size	(2, 2)
Learning rate	0.0001	Batch size	32
Validation split	0.2	Activation function	ReLU
Smart optimization	Talos hyperparameter	Filter size	5^*∗*^5
Dropout rate	0.5	Padding	SAME
Epochs	50		

**Table 3:** Datasets descriptions.

Datasets	Image size	#Classes	#Training sets	#Testing sets
DS1 [38]	512^*∗*^512	2	15264	400
DS2 [37]	1024^*∗*^1024	3	1811	484

**Table 4:** DeepLabv3plus training parameters.

Parameters	Values
Input size	256^*∗*^256
Learning rate	0.001
Epochs	30
Activation function	SoftMax
Batch size	10

**Table 5:** Results of experiments on DS1 using (RESNET-50+ DenseNet) and binary classifier.

	Without data augmentation (%)	Without semantic segmentation (%)	Without pruning (%)	Full features (%)
Sensitivity	90.57	93.34	96.90	99.6
Specificity	88.43	91.23	94.33	98.9
Accuracy	89.03	92.59	95.88	99.6
*F*1-score	89.20	92.70	95.90	99.6

The article "COVID-19 Semantic Pneumonia Segmentation and Classification Using Artificial Intelligence" was retracted in 2025. Reasons: signs of a paper mill; suspected computer-generated content; unreliable results or conclusions; concerns about the data.

**Table 6:** Results of experiments on DS2 using (RESNET-50+ DenseNet) and multilabel classifier.

	Without data augmentation (%)	Without semantic segmentation (%)	Without pruning (%)	Full features (%)
Sensitivity	92.37	95.20	97.80	99.5
Specificity	90.63	94.80	95.43	99.1
Accuracy	91.13	95.11	96.62	99.6
*F*1-score	91.15	95.09	96.80	99.6

**Table 7:** Comparison between proposed model and related works.

N	Ref.	Model techniques	Average accuracy	Running time (min)
1	[15]	Truncated inception network	98.5	110
2	[16]	DarkCovidNet	87.02	-
3	[9]	Bayes-SqueezeNet	97.9	-
4	[17]	DenseNet	85	
5	[18]	MobileNet	94.7	40
6	[19]	Resnet-50 + SVM	94.7	52
7	[20]	CXRVN	97.5	45
8	[33]	Weighted average pruned	98.1	38
9	Our model	Semantic segmentation + (ResNet 50 and DenseNet) + weighted average pruned	99.6	48

## Data Availability

All data used to support the findings of the study are included within the article.
